The article "The potency of natural resources and trade globalisation in the ecological sustainability target for the BRICS economies" was retracted in 2025. Reasons: unreliable results or conclusions; concerns about the citations.

# The potency of natural resources and trade globalisation in the ecological sustainability target for the BRICS economies

**DOI:** 10.1016/j.heliyon.2023.e15734

**Published:** 2023-04-25

**Authors:** Tomiwa Sunday Adebayo, Ahmed Samour, Andrew Adewale Alola, Shujaat Abbas, Mehmet Ağa

**Affiliations:** a Department of Economics, Faculty of Economic and Administrative Science, Cyprus International University, Nicosia, Northern Cyprus, via Mersin-10, Turkey; b Department of Accounting , Dhofar University, Salalah, Sultanate of Oman; c CREDS-Centre for Research on Digitalization and Sustainability, Inland Norway University of Applied Sciences, Norway; d Faculty of Economics, Administrative and Social Sciences, Nisantasi University, Istanbul, Turkey; e Graduate School of Economics and Management, Ural Federal University, Russian Federation; f Department of Accounting and Finance, Faculty of Economic and Administrative Science, Cyprus International University, Nicosia, Northern Cyprus, via Mersin-10, Turkey

**Keywords:** Ecological footprint, Natural resources, Renewable energy, Trade globalisation

## Abstract

The BRICS nations have yet to significantly contribute to achieving Sustainable Development Goals (SDG) 7 and 13. Dealing with this problem might necessitate a policy shift, which is the main topic of this research. Therefore, the current study scrutinizes the interrelationship between natural resources, energy, trade globalisation and ecological footprint using panel data from the period between 1990 and 2018 for the BRICS nations. To assess the interrelationship between ecological footprint and its determinants, we used the Cross sectional autoregressive distributed lag (CS-ARDL) and common correlated effects. mean group (CCEMG) estimators. The findings show that economic progress, and natural resources lessen ecological quality, while renewable energy and trade globalization improves ecological quality in the BRICS nations. Based on these results, the BRICS nations need to upgrade their use of renewable energy sources and improve the structure of their natural resource endowments. Furthermore, trade globalisation necessitates immediate policy responses in these nations since it reduces ecological damage.

## 1 Introduction

Balance is needed regarding developing and advanced economies' economic and environmental goals. The recent rapid growth in global economies has permitted them to alleviate poverty, build basic infrastructure, and enhance individuals' standard of living. On the other hand, in the quest for a fast economic boom, world economies have undermined natural capital, causing significant ecological problems such as biodiversity loss, energy resource extraction, land deterioration, and water and air contamination [1,2]. This issue, combined with increased human energy use, raises the vulnerability of humanity and exacerbates the planet's ecological resource shortage. Global product manufacturing and energy use reportedly account for 25% of global environmental emissions [3]. Consequently, failing to meet the Sustainable Development Goals (SDGs) will cause a massive ecological deficit as a result of the failure to create sustainable communities and reduce emissions [4,5]. The main objective is to accomplish economic progress while maintaining ecological integrity by reconciling human needs with the planet's regeneration capacity and exploring more environmentally-friendly approaches to avert socio-ecological crises.

Examining how natural resources affect the ecological footprint is the research's second goal. Woods, cropland, developed land, grazing land and fishing grounds are just a few examples of eco-friendly ecological footprint natural resources that help offset human-sourced CO_2_ and ease capital input for energy production [6,7]. On the other hand, many conventional natural resources, such as gas, petroleum products and coal, negatively impact the environment [8]. Nevertheless, natural resources are closely related to an economy's real income level. People overuse energy resources like natural resources in the early stages of the economic growth process while ignoring the environmental costs [9,10]. Nonetheless, preserving a healthier ecosystem, safeguarding natural resources, and using energy-efficient products becomes increasingly important as economic expansion moves into its later stages and people's living standards improve. In this sense, accelerating economic expansion will result in the increased exploitation of natural resources, industrial output, and agricultural outputs, all of which will expedite the depletion of natural resources [11].

Parallel to this, globalisation has intensified in most nations in recent decades, having beneficial and harmful effects on different fronts [[12], [13], [14]]. The importance of geography has diminished as social, political and economic connection has expanded between nations that share borders. The underlying principles of globalisation promote trade in services and goods, which has a direct and indirect effect on the contamination of the environment. On the other hand, evidence suggests that globalisation fosters the deployment of more sustainable production methods and accelerates the transfer of technologies [15,16]. Other study findings indicate that the ecological impact of globalisation is varied in terms of contamination [13,16]. When multiple measurements of globalisation are applied, the findings are very disparate. Conversely, empirical research linking knowledge to ecological quality indicates that the interrelationship between the two indicators is advantageous for ecological sustainability [12,14,17]. The empirical evidence is generally insufficient to draw concrete conclusions about how globalisation affects the environment.

Early research on environmental destruction has tried to attribute CO_2_ as a major cause of the issue, while [18] claimed that CO_2_ only plays a minimal role in ecological issues. By deforestation, the purchase of agricultural land, and mining [19,20] also indicate that using NR for economic operations creates CO_2_, but it is not the only factor determining ecological damage. Scholars thus require a comprehensive indicator that can address the bigger issue. In this regard, the scholars utilized ecological footprint (EF) to measure environmental deterioration [3,21]. According to Refs. [6,22], ecological footprint is a proxy that measures the ability of biologically productive water and land to replicate all the resources of society and infuse their waste. Additionally, in an ongoing effort to attain economic development and growth, countries are consuming increasing amounts of natural resources, which is widening the ecological deficit.

The biological capability for output must be greater than the ecological demand from consumption for sustainable development to be accomplished. Energy structure is nevertheless crucial considering the current economic climate and rent on natural resources. Regarding overall energy usage, renewable energy sources comprise a portion of the energy structure [23,24]. Switching to renewable energy sources is desirable because it is considered an environmentally-friendly alternative [25]. Additionally, the literature extensively discusses how renewable energy can help reduce ecological footprints. The previously mentioned information motivated us to formulate the research objectives by asking the basic questions: (a) Do economic growth and fossil fuel contribute to the ecological footprint of the BRICS nations? (b) What is the role of natural resources on the ecological footprint of the BRICS economies? (c) How does renewable energy decrease ecological footprint in the BRICS nations? (d) Does trade globalization decrease EF in the BRICS nations?

The BRICS nations account for 26% of global GDP as well as 41% (see Fig. 1) of worldwide CO_2_ [26]. India, Russia, Brazil and China are among the top seven countries on the planet for CO_2_ [26]. Compared to the developed countries, the BRICS face far more severe ecological concerns. This is because, between 1990 and 2018, CO_2_ in the BRICS increased from 27 to 42%, while CO_2_ in the EU countries declined from 40 to 25% [26]. Considering that the BRICS enjoyed annual growth of 6.5% (on average) over the last ten years, these emerging countries must modernise their current technologies and create new cutting-edge technology to lessen harmful development externalities.

**Fig. 1:** Information on BRICS nations.

In this regard, it is essential to give the issue of ecological degradation in the BRICS region additional attention; otherwise, the growing threats and hazards linked with global warming in the coming years will have a disastrous effect on human well-being. Additionally, there is a substantial vacuum in the past empirical research in terms of estimating impact of trade globalisation, renewable energy, and fossil fuels on ecological footprint. As a result, we used ecological footprint, a broader measure of environmental deterioration, to evaluate the effect of fossil fuel, renewable energy, and trade globalisation on ecological footprint. Last but not least, second-generation econometric techniques were used in this investigation since they are capable of addressing a number of methodological issues such as endogeneity, normality, and the capacity to explain a wider range of changes than traditional statistical techniques. Additionally, second-generation approaches are recognized as sophisticated, valid and reliable for handling panel data sets, particularly in the context of cross-sectional dependence and heterogeneity.

Following that, the remaining research components are divided into four segments: a synopsis of past studies is presented in Section 2. The technique and data are presented in Section 3, while the interpretations of the results are found in Section 4. The research's ramifications and policy framework are discussed in Section 5.

## 2 Synopsis of studies

The main issue confronting mankind is global warming and climate change, which result from increased environmental degradation caused by various human activities. As a result, several international bodies, policymakers, and scholars have highlighted the importance of climate change and global warming mitigation. Such initiatives can be seen in COP21 in Paris, COP 26 in Glasgow and COP 27 in Sharm El-Sheikh. The motives of the gathering are to reaffirm each nations commitment to cutting CO_2_ emissions and their path towards carbon neutrality targets. Over the years, scholars mostly in the domain of energy and environmental economics have explored the role of economic variables such as financial development, globalization, disintegrated energy, natural resources and economic growth on environmental degradation/quality proxies (CO_2_ emissions, ecological footprint, N_2_O, carbon footprint, and biocapacity etc.). However, inconclusive results have emerged regarding these connections, which can be attributed to the methods employed, time-period of investigation, and nation/nations of study.

### 2.1 Economic growth, renewable energy, and environmental degradation

The various international gathering on climate change and global warming have highlighted the energy transition from fossil fuel-based to renewables as the solution to climate change. Several studies have documented the decreasing emissions role of green energy, which is eco-friendly as the solution for mitigating environmental degradation. Significant empirical studies in the existing literature have demonstrated that renewable energy (REC) mitigates ecological deterioration. For instance Ref. [27], explored the role of REC in carbon mitigation for the case of 15 selected economies, and their study finding disclosed that carbon reduction is achieved in 15 selected economies via the use of REC. Likewise, the studies of [28] on the role of green energy towards carbon reduction in India using the non-linear approach disclosed that positive (negative) changes in green energy lessen carbon emissions in India. Likewise, for the case of United States (US) [29], documented the emissions-lessening role of renewable energy within the framework of the EKC hypothesis. Likewise, in the case of France [30], research documented that carbon decrease can be achieved via using sustainable energy. The study of [30] is also backed by the study of [31] on the case of France, who documented that the intensification of renewable energy caused a lowering of ecological deterioration. Meanwhile [32], revealed that REC in BRICS nations mitigates environmental degradation from 1992 to 2018. Using the CS-ARDL technique [33], tested the impact of REC on the ecological environment in sovereign Nordic countries. The results show a significant interconnection between REC and ecological integrity that is found to be beneficial. Recently [34], argued that REC significantly influenced environmental neutrality in the case of BRICS states from 1990 to 2019.

The motive of all economies is to achieve economic growth; however, most of these countries achieved this growth at the expense of ecological sustainability. Thus, it is important for nations to switch to sustainable growth. In this line, several studies have reported various dimensions regarding the linkage between growth and ecological sustainability/deterioration. For instance Ref. [35], in China's case reported that China's economic growth is not sustainable as an increase in real GDP intensifies CO_2_ emissions. Similar result is also documented by the study of [36] for OECD, which highlighted the emission-increasing role of economic expansion. Likewise [37], evaluated the emissions-growth nexus in the USA using the bootstrap Granger causality with the result suggesting that growth in the USA is not sustainable. The studies of [38]also document the ecological deterioration increasing role of economic expansion [22] for the BRICS economies and [39] for BRICS [40] for Turkey. In the same vein, the study of [41] using the FMOLS on the linkage between growth and emissions affirmed the EKC hypothesis, which stipulates the increasing economic growth role in the initial phase of development while emissions decreasing role of economic growth is observed in the second phase.

### 2.2 Natural resources and environmental degradation

The interconnections between natural resources and ecological quality have received scholars' attention over the last few years. Some empirical studies found that natural resources promote ecological quality: For instance Ref. [6],confirmed that a significant increase in natural resources contributed to reducing ecological degradation in the USA from 1980 to 2017. Recently [42], showed that natural resources negatively influences ecological pollution in G7 nations from 1990 to 2020. In contrast, some studies found natural resources mitigate environmental sustainability. For example [43], showed that natural resources positively affected ecological pollution in the BRICS states from 1996 to 2018. Likewise [44], employed the method of ARDL and suggested that an improvement in ecological quality in the USA is attributed to a significant increase in natural resources. On the other hand, some researchers found no significant interconnection among the mentioned variables. For example [45], showed no significant effect of natural resources on carbon (CO2) emissions in the BRIC states from 1990 to 2015. Recently [46], also argued that the interconnection between natural resources rent and EF in seven emerging countries is insignificant.

### 2.3 Globalization and environmental degradation

Scientific studies have thoroughly documented the interconnection between globalization and environmental degradation. Some of the empirical studies emphasized that globalization mitigates ecological degradation. For example [47], assessed this relationship in the high- and middle-income economies and highlighted that a rise in globalization mitigated environmental degradation for the time from 19970 to 2012 [48]. further argue that globalization mitigates the ecological quality in Argentina for the time from 1970 to 2018 [49]. additionally assessed the same relationship for the BRICS economies. The outcomes suggest that globalization promotes ecological integrity between 1990 and 2017. Moreover [50], also examined a similar linkage and region from 1990 to 2019. Apart from discovering globalization has a significant influence on ecological integrity [51]. confirmed a positive interrelationship between globalization and ecological integrity of the BRICS economies from 1990 to 2018. The recent research conducted by Ref. [52] in the BRCIS-T states reported that globalization significantly helps reinforce ecological integrity over the period of analysis from 2000 to 2020. In contrast, few studies emphasized that globalization's adverse influence on the ecological proxies, implying that globalization mitigates environmental quality. For example [53], assessed the same relationship in the BRIC economies from 1971 to 2016. The author showed that globalization mitigates the ecological integrity in the tested economies [54]. further argue that globalization alleviates environmental neutrality in the case of G7 nations from 1996 to 2017.

### 2.4 Fossil fuel and environmental degradation

Numerous studies have explored the interconnection between fossil fuel consumption (FF) and environmental degradation. For instance Ref. [55], assessed the interconnection among fossil fuel and CO_2_ emissions for 19 selected nations from 1990 to 2014. The findings showed that fossil fuel mitigates environmental integrity. Moreover [56], reported a positive interconnection between fossil fuels and ecological degradation. The authors suggest that policymakers in the BRICS must put more effort into promoting green energy to reinforce environmental quality in BRICS nations. Similarly [57], examined a similar interconnection for BRICS nations from 1990 to 2017. Apart from discovering fossil fuel has a negative influence on ecological integrity. Findings showed that fossil fuel mitigates the ecological integrity in the tested countries [58]. also found that fossil fuel surged ecological pollution in BRICS from 1995 to 2015 [59]. demonstrated that fossil fuels led to an increased ecological footprint in India [41]. suggest that an augmentation in fossil fuel mitigates the ecological integrity in the BRICS states from 1990 to 2018. Moreover [60], recently showed that fossil fuel mitigates ecological quality in the BRICS states from 1990 to 2018 [61]. analyzed fossil fuel and the ecological pollution of the BRICS countries from 2003 to 2018. The authors suggested that the surge in environmental pollution in BRICS is attributed to a rise in fossil fuel.

## 3 Data and empirical methodology

### 3.1 Model and data

The current investigation explores the influence of NR, FF, TGLO, GDP and REC on the EF in BRICS countries. In doing so, we employed annual data covering 1990–2018. The dependent variable is EF which represents ecological footprint. The independent variables are REC which represents renewable energy, TGLO represents trade globalisation, NR denotes natural resources and GDP stands for economic growth. To ensure the variables align with normality, we took the natural log of the series, which is in line with the studies of [[62], [63], [64]]. The economic model of the study is presented in Equation (1) as follows:

(1) $$\ln\;{EF}_{it}=\mu_{0}+\mu_{1}\;\ln\;{GDP}_{it}+\mu_{2}{lnREC}_{it}+\mu_{3}{lnNR}_{it}+\mu_{4}{lnFF}_{it}+\mu_{5}{lnTGLO}_{it}+\varepsilon_{it}$$

Where $\ln\;{EF}_{it}$, $\ln\;{GDP}_{it}$, ${lnREC}_{it}$, ${lnNR}_{it},{lnFF}_{it},{TGLO}_{it}$ represent ecological footprint, economic progress, renewable energy consumption, natural resources, fossil fuel consumption, and globalization, respectively. The variables, measurements, and data sources are reported in Table 1. Besides, Fig. 2a, Fig. 2ba and b presents the investigation series' scatter and box plots.

**Table 1:** The variables, measurement, and sources of data.

Sign	Variable	Measurement	source
EF	Ecological footprint	Per capita, global hectares	Global Footprint Network Database
NR	Natural resources	% of GDP.	World Bank Database
REC	Renewable energy consumption	Terawatt-hours (TWh).	Ourworldindata Database
GDP	Economic growth	Per capita (Constant-2015 US$).	World Bank Database
TGLO	Trade Globalization	Index	KOF database
FF	Fossil fuel consumption	Terawatt-hours (TWh).	Ourworldindata

**Fig. 2a:** Scatter plot of variables.

**Fig. 2b:** Box Plot of the series.

### *3.2* Econometric methodology

#### 3.2.1 Panel unit root and cross-sectional dependence

The checking of cross-sectional dependence (CD) is compulsory before running the unit root assessments. This CD assessment guides the scholars on whether to go for the first or second-generation tests. Therefore, the CD test proposed by Ref. [65] is employed to check the cross-sectional issue for each examined variable (Eq (2)).

(2) $$CD=\sqrt[{.}]{\frac{2T}{N\left(N-1\right)}}\left(\sum_{i=1}^{n-1}.\sum_{K=i+1}^{N}p_{IK}\right)\;N\left(0,1\right)I,K=1,2,3,\ldots \ldots \ldots N$$

where N stands to the cross-sections; T refers to time. To check the slope heterogeneity issue, the study uses the homogeneous assessment suggested by Ref. [66]. In this test, the $H_{0}$) is homogeneous, and $H_{1}$ is not homogeneous. The equations for checking the slope heterogeneity assessments are as follow:

(3) $${\tilde{\Delta }}_{SH}={\left(N\right)}^{\frac{1}{2}}{\left(2k\right)}^{-\frac{1}{2}}\left(\frac{1}{N}\tilde{S}-k\right)$$

(4) $${\tilde{\Delta }}_{ASH}={\left(N\right)}^{\frac{1}{2}}{\left(\frac{2k(T-k-1}{T+1}\right)}^{-\frac{1}{2}}\left(\frac{1}{N}\tilde{S}-2k\right)$$

In addition, the study employs the second-generation cross-sectional augmented Im–Pesaran–Shin (CIPS) assessment as advanced by Ref. [67] and Covariate, Augmented Dickey-Fuller (CADF) as advanced by Ref. [68] to evaluate levels of stationary amid the studied variables. These assessments are preferred over first-generation unit-root assessments because they consider the heterogeneity and cross-sectional dependence issues. The test statistic of CADF assessment, which is estimated on CIPS, is formulated as follows:

(5) $$\hat{CIPS}=\frac{1}{N}\sum_{i=1}^{n}{CADF}_{i}$$

#### 3.2.2 Co-integration testing

To capture the long-term co-integration among the focused variables, the research uses co-integration approaches suggested by Ref. [69]. In comparison with classical tests of co-integration, these tests have more advantages than classical co-integration tests because of their features to tackle CSD, stationary, and heterogeneity. The Westerlund assessment developed into four tests, which are formulated as follows:

(6) $${Gt}_{test}=\frac{1}{N}\sum_{i=1}^{N}\frac{{\hat{\alpha }}_{i}}{C.S.E\left({\hat{\alpha }}_{i}\right)}\text{.}$$

(7) $$G_{\alpha }\;tests=\frac{1}{N}\sum_{i=1}^{N}\frac{T{\hat{\alpha }}_{i}}{\left({\hat{\alpha }}_{i}\right)\left(1\right)}\text{.}$$

(8) $${Pt.}_{test}=\frac{{\hat{\alpha }}_{i}}{CSE\left({\hat{\alpha }}_{i}\right)}$$

(9) $$P_{\alpha \;test.}=\frac{T{\hat{\alpha }}_{i}}{\left({\hat{\alpha }}_{i}\right)\left(1\right)}$$

In this test, $H_{0}$ assumes no co-integrating linkage among the focused variables. While $H_{1}$ assumes that there is a co-integrating linkage among the focused variables.

#### 3.2.3 CS-ARDL test

To evaluate the linkage among GDP, globalization, REC, FF, natural resources, and ecological footprint; the work utilizes the upgraded approach of cross-sectionally augmented autoregressive distributed lags (CS-ARDL). Classical methods, such as random and fixed effects, disregard cross-sectional dependence, which may lead to incorrect outcomes [70]. To overcome this issue, this work utilizes the upgraded approach of the CSARDL. However, the CSARDL model has some advantages over other traditional methods. For example, this model provides robust findings even as the variables are integrated by I (0)/(1) or both. In addition, this approach can give precise outcomes in the occurrence of short and long-run CSD. The baseline of the CSARDL estimation is formulated as follow:

(10) $$y_{it}=\beta_{i}+\sum_{l=1}^{P}\vartheta_{1i}y_{i,t-1}+\sum_{l=0}^{q}\emptyset_{1i}X_{i,t-1}+\sum_{l=0}^{q}\varphi_{1,i}\bar{Z_{i,t-1}}+\varepsilon_{it}$$

In Eq. (10), $\bar{Z_{i,t-1}}$ −l refers to lagged cross-sectional averages $\bar{Z_{i,t-1}}$ = ($y_{i,t-1},X_{i,t-1})$. q means lag options for the averages of the cross-section. $\varepsilon_{it}$ stands the error, the long-run coefficients will be captured employing the pooled mean group approach, which is given below as:

(11) $$\hat{\pi }=\frac{\sum_{l=0}^{q}{\hat{\emptyset }}_{il}}{1-\sum_{l=1}^{p}{\hat{y}}_{il}}$$

where $\hat{\emptyset }$ stands individual estimations for each cross-section. However, the error correction (ECM) form of the CS-ARDL approach is given below as:

(12) $${\Delta y}_{it}=\beta_{i}\;\left[y_{i,t-1}-\theta x_{i,t-1}\right]-\sum_{l=1}^{P}\vartheta_{1i}y_{i,t-1}+\sum_{l=0}^{q}\emptyset_{1i}X_{i,t-1}+\sum_{l=0}^{q}\varphi_{1,i}\bar{Z_{i,t-1}}+{\omega_{it}+\varepsilon }_{it}$$

where ω denotes error correction speed of adjustment. The error correction mechanism in CS-ARDL means that the tested economies are approaching equilibrium.

#### 3.2.4 Robust models

In addition, the current work utilized the augmented mean group approach (AMG), and the common correlated effect mean group approach (CCEMG) to assess the reliability of the CS-ARDL testing model for robustness. These tests also are considered consistent and efficient. AMG test equation in the first and second stages are formulated as follow:

(13) $$y_{it}=\delta_{i}\Delta_{Xit}+\alpha_{i}\sum_{I=2}^{T}\text{,}D_{it}+\varepsilon_{it}$$

(14) $$y_{it}=\alpha_{i}+\delta_{i}\Delta_{Xit}+c_{i}t+D_{i}{\hat{\upsilon }}_{t}{+\varepsilon }_{it}$$

$y_{it}$ represents the dependent variable in the tested model, $X_{it}$ is the vector of explanatory variables, and $X_{it}$ the cross-sectional averages for $X_{it}$, where $f_{t}$ represents the unobserved common factor. Similarly, the mean group estimations can be captured as follows:

(15) $$AMG=N^{-1}\sum_{i=1}^{N}\text{,}{\tilde{\delta }}_{i}$$

where $\hat{\delta }$ i stands for OLS regression estimates of sector-specific coefficients as represented in equation (13).

CCEMG approach upgraded by Ref. [71], which is robust to both slope heterogeneity, structural breaks, and cross-sectional dependence. CCEMG approach equation is formulated as follows:

(16) $$Y_{it}=\alpha_{i}+\delta_{i}X_{it}+\beta_{i}\bar{Y_{it}}+\beta_{i}\bar{X_{it}}+{\beta_{i}\;f}_{t+}\varepsilon_{it}$$

(17) $$CCEMG=N^{-1}\sum_{i=1}^{N}\text{,}{\hat{\delta }}_{i}$$

$Y_{it}$ stands the dependent variable in the focused model, $X_{it}$ denotes the vector of repressors, where $\bar{X_{it}}$ the cross-sectional averages for $X_{it}$, where $f_{t}$ represents the unobserved common factor. Fig. 3 presents the flow of the study based on the techniques employed

**Fig. 3:** Flow of the analysis.

## 4 Findings and discussion

### 4.1 Pre-estimation test outcomes

We commence by presenting brief information of the data utilized in this empirical analysis. Table 2 presents descriptive statistics of the series of investigation. The outcomes show the values of standard deviation, median, minimum, mean and maximum, enabling enhanced comprehension of the data and how it is dispersed across the structure.

**Table 2:** Descriptive statistics.

	LnGDP	LnFF	LnEF	LnNR	LnREC	LnTGLO
Mean	7.9440	8.2524	0.9409	1.4186	5.5169	3.7245
Median	8.1514	8.2851	1.0878	1.3383	6.2016	3.7429
Maximum	9.6787	10.400	1.9222	3.0915	8.4628	4.2753
Minimum	5.7076	6.7209	−0.2727	−0.0522	−0.8399	2.9122
Std. Dev.	1.0871	1.0442	0.5996	0.7309	2.0835	0.3171
Skewness	−0.5270	0.3200	−0.6751	0.4194	−1.2707	−0.4850
Kurtosis	2.2555	2.0027	2.4315	2.6416	3.4473	2.8816

To find the suitable unit root test, we evaluate the CD test. The findings of the CD test are presented in Table 3. The results of the test statistics show that CSD appears in the BRICS nation's sample. Therefore, the null hypothesis of “no CSD” is dismissed at a 1% level of significance. The outcomes display proof of CSD in GDP, FF, REC, NR and TGLO. We use the [72] CADF and CIPS unit root tests after validating the occurrence of CSD. In addition to checking for unit root, both tests give information regarding the series' heterogeneity. The unit root surface for all series (see Table 4). At the first difference, nevertheless, all series are noticeably stationary.

**Table 3:** CD and CIPS and CADF test outcomes.

Variables	CD Outcomes	*p-value*	CIPS Outcomes		CADF Outcomes	
			*I(0)*	*I(I)*	*I(0)*	*I(I)*
LnEF	11.891***	0.000	−1.893	−4.508***	−1.631	−4.280***
LnGDP	6.0206***	0.000	−0.481	−4.305***	−2.250	−3.539***
LnREC	10.103***	0.000	−2.269	−4.261***	−2.241	−4.750***
LnTGLO	8.4683***	0.000	−0.585	−4.337***	−1.574	−3.149***
LnFF	10.937***	0.000	−1.383	−3.948***	−1.738	−4.394***
LnNR	9.8962***	0.000	−1.873	−5.605***	−2.479	−4.133***

**Note:** ***P<1%.

**Table 4:** Slope heterogeneity test.

$\hat{\Delta }$	P-value	${\hat{\Delta }}_{Adj}$	P-value
5.580***	0.000	6.407***	0.000

Note: ***P<1%.

The slope heterogeneity assessment as presented in Table 4. The findings illustrated that both $\hat{\Delta }\;and\;{\hat{\Delta }}_{Adj}$ reject the null hypothesis of slope homogeneity at 1% significance level. Thus, the explored model specification in this work is correct.

### 4.2 Cointegration results

It is crucial to evaluate the existence of cointegration amongst the investigation parameters. In doing so, we employed Panel cointegration methods suggested by Refs. [69,73] to explore the interrelationship between EF and the regressors for the BRICS nations. The [69] cointegration results dismissed the null hypothesis of “no cointegration,” as revealed in Table 5. This shows an interrelationship between LCF and economic growth, renewable energy consumption, banking development, and natural resources for the BRICS nations in the long run.

**Table 5:** Westerlund cointegration outcomes.

Statistics	Value	Z-value	*p*-value	Robust P-value
Gt	−3.711	−1.691	0.045	0.000
Ga	−12.636	1.607	0.946	0.000
Pt	−7.776	−1.553	0.060	0.000
Pa	−14.748	0.231	0.592	0.000

### 4.3 CS-ARDL results

The current investigation employed the CS-ARDL to evaluate the association between EF and the explanatory variables, the results of which are illustrated in Table 6. The ECT is predicted to have a significant negative effect, implying that the system returns to a long-term equilibrium following a shock. This procedure, as stated previously, shows the existence of cointegration among the series.

**Table 6:** CS-ARDL results.

	Long-run Results			
	Coefficients	SE	Z-statistics	Pvalue
LnGDP	0.0640***	0.0143	4.46	0.000
LnNR	0.0256**	0.0104	2.44	0.015
LnTGLO	−0.0390***	0.0100	−3.90	0.000
LnFF	0.1821***	0.0391	4.63	0.000
LnREC	−0.0476***	0.0177	−2.68	0.007
	Short-run Results			
LnGDP	0.1195***	0.0240	4.98	0.000
LnNR	0.0478**	0.0190	2.50	0.012
LnTGLO	−0.0831	0.0569	−1.46	0.144
LnFF	0.3578***	0.0861	4.15	0.000
LnREC	−0.0903***	0.0321	−2.81	0.005
ECT (-1)	−0.9042***	0.0909	−9.94	0.000

**Note:** ***P<1%, **P<5%, and * P<10%.

The positive effect of economic growth on EF is observed in both the long and short run. This suggests that the scale effect dominates the composition and technique effects in the BRICS economies. Economic activity has expanded due to economic expansion, including the industrialization of all aspects of their economies and the exploitation of natural resources. The ecological condition has decreased and EF levels have risen as a result. All economic actions are ecologically motivated since the environment and development are closely related. The economic growth rate witnessed by the BRICS countries over the preceding two decades provides another reason for GDP's effect on improving EF. Recent arguments suggest that industrial expansion has damaged ecological integrity despite being economically attractive. The unpredictable emissions levels in the BRICS countries have deteriorated due to more industrial operations and economic expansion. The studies of [18,74] for Finland, and [75] for China reported similar results.

As expected, the effect of FF on EF is significant and positive. These results were predicted given that fossil fuels add to global warming by producing energy and generating CO_2_ and other greenhouse gases (GHGs) when consumed. According to the findings, the BRICS governments should concentrate on shifting away from fossil fuels, which contribute to growing emissions, and toward more affordable and trustworthy clean energy sources supporting a stable climate and sustainable growth. Additionally, more government funding should be allocated to investigate and create fresher solutions to the nation's ecological problems. The BRICS government's increased investment in R&D would improve the efficiency of the production of energy resources and encourage FDI capital inflows into their economies. The BRICS countries may achieve their SDGs by reducing emissions by switching from fossil fuels to green energy. The studies of [25] for BRICS [32], for BRICS [76], for Russia and [77] documented similar findings.

As anticipated, a decrease in EF is caused by an intensification of REC in the BRICS nations. This demonstrates that an upsurge in REC promotes ecological quality in the BRICS nations. This shows that switching to more ecologically friendly or ecologically conscientious energy sources provides benefits to the ecosystem. This is compatible with from the findings of several earlier investigations [31,51,56]. However, the findings contradict the studies of [75,78,79], which documented the emission increasing role of renewable energy.

In addition, we found a negative link between trade globalization and EF. This result demonstrates that the BRICS countries have stronger emissions reductions due to the trend toward trade globalization. For the BRICS nations, the results supported the pollution halo hypothesis (PHH). The studies of [14,80,81] also affirmed the pollution halo hypothesis. However, the studies of [13,16,82] refute our findings by affirming the pollution haven hypothesis. Additionally, we observed a favorable natural resource-EF linkage, which shows that natural resources lower environmental quality. This depicts how the depletion of natural resources negatively impacts the BRICS countries' environmental quality. This outcome complies with the works of [10,11,21,83].

#### 4.3.1 Robustness check with CCEMG

We used the CCEMG estimator to evaluate the reliability of the CS-ARDL approach (See Table 7). The results revealed that FF, GDP and NR contribute to decreased ecological quality while REC and TGLO contribute to an upsurge in ecological quality in the BRICS nations. Fig. 4 presents a summary of findings from the CS-ARDL and CCEMG estimators.

**Table 7:** Robustness check with CCEMG.

	Coefficients	SE	Z-statistics	Pvalue
LnGDP	0.0628**	0.0264	2.38	0.017
LnNR	0.0817***	0.0265	3.072	0.000
LnTGLO	−0.0955**	0.0402	−2.25	0.018
LnFF	0.4768***	0.0810	5.88	0.000
LnREC	−0.0393***	0.0131	−2.99	0.003

**Note:** ***P<1%, **P<5%, and * P<10%.

**Fig. 4:** Summary of findings from CS-ARDL and CCEMG

#### 4.3.2 Panel causality results

This research used the panel causality test to investigate the causal connection among variables of investigation. Table 8 presents the causality results and we observed that all the series could predict ecological deterioration. These outcomes correspond with the prior studies.

**Table 8:** Panel causality results.

Dependent Variables	Independent Variables					
	LnEF	LnGDP	LnNR	LnTGLO	LnFF	LnREC
LnEF		5.857***	2.609***	3.139***	6.863***	2.791***
LnGDP	3.719***		3.751***	6.002***	8.498***	0.743
LnNR	0.964	0.620		2.028**	1.886	1.063
LnTGLO	0.173	1.279	5.299***		1.519	1.132
LnFF	1.520	2.735***	1.745	7.773***		3.601***
LnREC	0.206	3.602***	0.353	1.793	4.526***	

**Note:** ***P<1%, **P<5%.

## 5 Conclusion and policy implications

### 5.1 Conclusion

The purpose of this study was to scrutinize the interrelationship between natural resources, energy and ecological footprint using panel data from the period between 1990 and 2018 in the BRICS nations. To do this, the research began the econometric evaluation by searching for CD in the data. After identifying CD in the series, we conducted the CIPS and CADF second-generation unit root tests, and all parameters were found to be I (1). Then, we investigated the long-run cointegration using the technique from Ref. [69]. To assess the relationship between the ecological footprint and its determinants, we used the CS-ARDL and CCEMG estimators. The findings showed that economic progress and natural resources lessen ecological quality while renewable energy and trade globalization improve ecological quality in the BRICS nations.

### 5.2 Policy remarks

The following policy remarks are highlighted in line with the conclusions drawn from the findings above.

➢ Environmental deterioration manifests in the BRICS countries as a result of both economic expansion and fossil fuel usage. The BRICS countries may face significant long-term ecological consequences due to their unsustainable fossil fuel usage in this climate. The researched countries should strive to divorce economic expansion from fossil fuel usage in order to avoid massive ecological costs. However, a complete decoupling may be unthinkable, considering that the BRICS countries are emerging economic giants and that doing so would push their economies into recession. In this situation, these nations might choose to decouple gradually by increasingly leaning toward renewable sources of energy. The researched countries may also evaluate whether adopting a green growth strategy will be feasible in the long run.
➢ The exploitation, processing, and use of natural resources may contribute to ecological problems such water, air, and land pollution, disturbance of ecosystems, and a reduction in biodiversity. In order to secure sustainable natural resource exploitation via environmentally friendly, scientific mining, the BRICS authorities must take major measures. Environmentally responsible mining discourages the overuse of ecosystem services, which aids in the recovery of biocapacity surplus. Furthermore, the governments of the BRICS should not overly depend on natural resources and instead focus on developing other industries that can substantially contribute to the creation of ecosystem services proxies that can aid in easing excessive environmental pressure. As was already established, one of the major environmental hazards in the BRICS group has been coal mining. As a result, the BRICS governments should gradually stop mining coal in favor of less-emitting fossil fuels like natural gas. The BRICS nations should also use the revenue they obtain from renting out their natural resources to invest in creating clean and renewable energy sources.
➢ There is a key lesson for the BRICS countries, particularly from the globalization standpoint: trade globalization significantly contributes to improving ecological quality. Thus, these nations' borders should be opened to other nations, particularly those already enforcing ecological standards for tradeable goods. Since individual markets are currently working on returning to a growth trajectory after the fallout and losses from the Covid-19 pandemic, the BRICS should embrace a more determined push towards creating an eco-friendly globe via low-carbon technologies investment and clean industrialization. The future lies in renewable goods and a sustainable economy. Hence. the shift to this new stage must be free of compromise and uncertainty regarding the dedication to taking action on climate change. Countries have pledged to achieve net-zero emissions by the middle of the century. Nevertheless, as observed by the UNEP (2021), this objective has thus far been hampered by setbacks brought on by political resistance and the inability to carry out strategies, amongst many other problems.

### 5.3 Limitation of study and future directions

The paper's drawback is that it merely examines the effects of trade globalisation on ecological footprint while the corresponding effects of other aspects of globalisation, such as financial, economic, and social globalization, are yet to be explored. Future research should thus examine these areas of study.

## Author contribution statement

Andrew Adewale ALOLA: Wrote the paper; Contributed reagents; Analyzed and interpreted the data.

Ahmed Samour: Wrote the paper, Materials, analysis tools, and data; Contributed reagents.

Tomiwa Sunday Adebayo: Wrote the paper, materials, analysis tools; analyzed and interpreted the data.

Mehmet Ağa: conceived and designed the analysis; Contributed reagents; Wrote the paper.

Shujaat Abbas: Analyzed and interpreted the data; Conceived and designed the analysis: Wrote the paper.

## Data availability statement

Data will be made available on request.

## Declaration of interest's statement

The authors declare no conflict of interest.
